The article "Prediction of Functional Genes in Primary Varicose Great Saphenous Veins Using the lncRNA-miRNA-mRNA Network" was retracted in 2023. Reasons: signs of a paper mill; compromised peer review; unreliable results or conclusions.

# Prediction of Functional Genes in Primary Varicose Great Saphenous Veins Using the lncRNA-miRNA-mRNA Network

**DOI:** 10.1155/2022/4722483

**Published:** 2022-09-08

**Authors:** Jiabo Wei, Haihong Zhu, Qijun Zhang, Qin Zhang

**Affiliations:** ^1^Vascular Surgery Department, The Affiliated People's Hospital of Ningbo University, Ningbo University, Ningbo, Zhejiang, China; ^2^Cardiothoracic Surgery Department, The Affiliated People's Hospital of Ningbo University, Ningbo, Zhejiang, China; ^3^Cardiovascular Department, The Affiliated People's Hospital of Ningbo University, Ningbo University, Ningbo, Zhejiang, China

## Abstract

**Background:**

Long noncoding RNAs (lncRNAs) have been widely suggested to bind with the microRNA (miRNA) sites and play roles of competing endogenous RNAs (ceRNAs), which can thus affect and regulate target gene and mRNA expression. Such lncRNA-related ceRNAs are identified to exert vital parts in vascular disease. Nonetheless, it remains unknown about how the lncRNA-miRNA-mRNA network functions in the varicose great saphenous veins.

**Methods:**

This study acquired the lncRNA and mRNA expression patterns from the GEO database and identifies the differentially expressed mRNAs and lncRNAs by adopting the R software “limma” package. Then, miRcode, miRDB, miRTarbase, and TargetScan were used to establish the miRNA-mRNA pairs and lncRNA-miRNA pairs. In addition, the lncRNA-miRNA-mRNA ceRNA network was constructed by using Cytoscape. Protein-protein interaction, Gene Ontology functional annotations, and Kyoto Encyclopedia of Genes and Genomes enrichment were carried out to examine the candidate hub genes, the functions of genes, and the corresponding pathways.

**Results:**

In line with the preset theory, we constructed ceRNA network comprising 12 lncRNAs, 38 miRNAs, and 149 mRNAs. Kyoto Encyclopedia of Genes and Genomes analysis indicated that the PI3K/Akt signaling pathway played a vital part in the development of varicose great saphenous veins. AC114730, AC002127, and AC073342 were significant biomarkers. At the same time, we predicted the potential miRNA, which may exert a significant influence on the varicose great saphenous veins, namely, miR-17-5p, miR-129-5p, miR-1297, miR-20b-5p, and miR-33a-3p.

**Conclusion:**

By performing ceRNA network analysis, our study detects new lncRNAs, miRNAs, and mRNAs, which can be applied as underlying biomarkers of varicose great saphenous veins and as therapeutic targets for the treatment of varicose great saphenous veins.

## 1. Introduction

Varicose veins, dilated, tortuous, and palpable veins, are the chronic venous disorder manifestations in clinic. Varicose great saphenous veins (GSVs) are particularly common and one of them [1]. The GSV incidence is predicted to be 10-20% and 25-33% among males and females, which also shows a rapidly elevating trend [2]. Age, sex, family history, and pregnancy account for the vital risk factors related to the formation of GSVs [3].

Valvular incompetence, hydrostatic pressure, and deep venous obstruction have been identified as the commonly seen characteristics of primary GSVs, which are identified as their etiology for a long time [4]. A number of molecules involved in numerous diverse pathways participate in diverse GSV-related pathological events, such as alterations of vascular structure and biochemical properties, the abnormal extracellular matrix, cytokine or growth factor imbalance, additional mechanisms, and genetic changes [2]. Nonetheless, these molecular mechanisms are just a part of the complicated mechanism network, so more studies should be conducted to explore the remaining mechanisms.

Noncoding RNAs are the RNAs that do not encode proteins and regulate gene expression at the transcriptional level, which include long noncoding RNAs (lncRNAs) and microRNAs (miRNAs) [5]. Of them, miRNAs represent the endogenous, single-stranded small ncRNAs that are 22-24 nucleotides in length [6]. miRNAs exert vital part in regulating different cell processes, such as growth, migration, differentiation, apoptosis, and metabolism [7]. In recent years, many articles report that lncRNAs exert vital parts in different diseases, including vascular diseases [8]. In addition, lncRNAs have been suggested to make interaction with miRNAs, thereby suppressing the degradation of target mRNAs via the regulating mechanism of competitive endogenous RNA [9].This lncRNA-miRNA-mRNA ceRNA network is suggested in certain disorders, but it has not been investigated in the context of GSVs. As a result, bioinformatic analysis should be performed to examine the ceRNA coregulation in GSVs, and this may help to establish a global regulatory mechanism and shed more lights on mechanisms of varicose great saphenous veins as well as the candidate therapeutic targets.

## 2. Materials and Methods

### 2.1. Data Collection

The GEO database (https://www.ncbi.nlm.nih.gov/geo/) can be used for next-generation sequencing of high-throughput microarray and international public functional genomics [10]. In the current work, the recently released gene expression profiles associated with GSVs were acquired from GEO (http://www.ncbi.nlm.nih.gov/geo). In addition, lncRNA and mRNA datasets were obtained from GSE51260 by adopting GPL15314 (Arraystar Human LncRNA Microarray V2.0 (Agilent_033010 Probe Name version)), which included 6 GSVs and 6 matched uninjured samples.

### 2.2. Differentially Expressed mRNAs (DEMs) and lncRNAs (DELs)

We use “Perl” language to convert probe matrix into gene matrix based on annotation information. Then, DEMs and DELs were detected between healthy subjects with GSV patients using the R software “limma” [11] package in accordance with the adjusted *P* < 0.05 and ∣log2(fold change) | >1 threshold. If log2(fold change) > 1, it indicates that this gene is upregulated in varicose veins group. If log2(fold change) < −1, it indicates that the gene is downregulated in varicose vein group.

### 2.3. lncRNA-miRNA-mRNA ceRNA Network Establishment

We selected the most significant GSV-associated lncRNAs from key modules for the prediction of miRNAs through miRcode (http://www.mircode.org) [12]. For constructing the ceRNA network, miRDB (http://www.mirdb.org/) [13], TargetScan (http://www.targetscan.org/) [14], and miRTarBase (http://mirtarbase.mbc.nctu.edu.tw//) [15] were adopted to predict miRNA target mRNAs. In addition, overlapped mRNAs and miRNAs, together with the corresponding interaction pairs, were applied in subsequent analyses. At last, the lncRNA-miRNA-mRNA network was established and visualized by Cytoscape (version3.6.1). Diverse shapes and colors were used to indicate 3 kinds of RNA types.

### 2.4. Gene Ontology (GO) and Kyoto Encyclopedia of Genes and Genomes (KEGG) Analyses

For further analysis, the DAVID Bioinformatics Resources 6.8 (https://david.ncifcrf.gov/tools.jsp) was employed for GO and KEGG pathway analyses on mRNA neighbors in the lncRNA-miRNA-mRNA network. DAVID can comprehensively explore the biological significance of numerous genes. A difference of *P* < 0.05 indicated statistical significance.

### 2.5. Protein-Protein Interaction Network and Hub Gene Analyses

To evaluate the relations of DEGs in ceRNA network, Search Tool for the Retrieval of Interacting Genes (STRING, https://string-db.org/) database was applied in the comprehensive analysis of interactions between proteins and genes, as well as the construction of the PPI network according to the as-constructed ceRNA network. Thereafter, Required Confidence (also referred to as the combined score) >0.4 was applied in visualizing the as-established PPI network [16]. The top 10 genes with the most adjacent nodes are chosen for further investigation using R software.

### 2.6. Critical lncRNA-miRNA-mRNA Subnetwork Reconstruction

This study obtained all lncRNAs and the corresponding mRNAs and miRNAs within the global triple-network for the construction of the novel subnetwork through adopting cytoHubba. Then, we determined the number of associated lncRNA-miRNA-mRNA triplets and screened target lncRNAs by the comparison between lncRNA node degrees and associated miRNA-mRNA and lncRNA-miRNA pair number.

## 3. Results

### 3.1. Selection of DELs and DEMs in GSV Patients

We acquired the lncRNA/mRNA expression profiles against GEO (GSE51260). After processing raw data, we discovered altogether 346 differentially expressed genes (DEGs) (Figure 1(a)). There were 46 DELs in the GSE51260 dataset, among which 42 were upregulated and 4 were downregulated (Figure 1(b)). At the same time, there were 300 DEMs, containing 86 upregulated and 214 downregulated ones (Figure 1(c)).

### 3.2. lncRNA-miRNA-mRNA ceRNA Network

Each miRNA is possibly related to multiple lncRNAs or mRNAs, whereas each lncRNA also possibly targets multiple miRNAs. According to the intersected elements, we discovered miRNA-mRNA and miRNA-lncRNA pairs. Therefore, this study constructed 38 miRNAs located in the ceRNA and constructed the ceRNA network. Thereafter, we established the lncRNA-miRNA-mRNA network comprising 12, 38, and 149 nodes of lncRNAs, miRNAs, and mRNAs, respectively. Cytoscape 3.5.1 was adopted for establishing the lncRNA-miRNA-mRNA ceRNA network (Figure 2).

### 3.3. GO and KEGG Analyses on DEMs in the ceRNA Network

GO and KEGG analyses were carried out by the DAVID tools to explore the mRNA functions within the constructed ceRNA network. mRNAs were discovered to be mostly enriched in the following terms: Wnt signaling pathway and negative regulation of MAP kinase activity in the “biological process” analysis (Figure 3(a)); in the “cellular component” analysis, many genes participated in nuclear, nucleoplasm, and nucleolus locations (Figure 3(b)); and protein binding in the “molecular function” analysis (Figure 3(c)). Meanwhile, as suggested by KEGG enrichment, some pathways were related to GSVs, such as the metabolic pathways and the PI3K-Akt signal transduction pathway (Figure 3(d)).

### 3.4. PPI Network Establishment and Key mRNA Verification

In order to further detect key mRNAs involved in the GSV-related ceRNA network, mRNAs in the ceRNA network were aligned against the STRING database. Besides, PPI network was established upon the threshold of comprehensive score > 0.4 (Figure 4(a)). The key mRNAs were chosen from the PPI network by applying the degree of linkage between DEMs. The top 10 key mRNAs with the highest degree of connectivity were discovered, including WDR3, SLU7, NCL, HNRNPR, SRSF4, HNRNPD, HELZ2, NUP133, PPIL4, and PIK3CA (Figure 4(b)).

### 3.5. Topology of GSV-Associated lncRNA-miRNA-mRNA Subnetwork

Hub nodes exert vital parts in the biological networks. As a result, for identifying hub RNAs as well as the corresponding networks, the node degrees related to ceRNA network were determined by the cytoHubba plug-in in Cytoscape. From ceRNA network, we found that there were three lncRNAs with more than 10 nodes (Table 1). lncRNA AC114730, lncRNA AC002127, and lncRNA AC073342 were the most significant nodes in the lncRNAs, which suggested that they exerted vital parts in gene modulation at transcriptional level. Thereafter, miRNAs and mRNAs related to the above 3 lncRNAs within the global triple-network were discovered, which were applied to reconstruct the novel subnetworks. Typically, the lncRNA AC114730-miRNA-mRNA network comprised 1, 19, and 96 nodes for lncRNAs, miRNAs, and mRNAs (Figure 5(a)); the lncRNA AC002127-miRNA-mRNA network comprised 1, 19, and 101 nodes for lncRNAs, miRNAs, and mRNAs, respectively, as well as 182 edges (Figure 5(b)). In addition, the lncRNA AC073342-miRNA-mRNA network comprised 1, 11, and 73 nodes of lncRNAs, miRNAs, and mRNAs, respectively, together with 114 edges (Figure 5(c)).

We predicted several important miRNAs through the principle of ceRNA network.  Table 2 presents the 10 most significant nodes with the highest degrees in the miRNA. Among them, the top five nodes are miR-17-5p, miR-129-5p, miR-1297, miR-20b-5p, and miR-33a-3p. Taking these miRNAs as the center, respectively, we built subnetwork (Figures 6(a)–6(e)).

## 4. Discussion

lncRNAs are associated with complicated effects achieved via different pathways, while ceRNA theory renders the most complex associations among mRNAs, lncRNAs, and miRNAs [17]. The present work adopted NCBI-GEO-derived interaction data for the generation of the global triple-network in line with ceRNA theory, suggesting that mRNAs and lncRNAs have identical miRNA within one triplet. Our constructed lncRNA-miRNA-mRNA network comprised 12, 38, and 149 nodes of lncRNAs, mRNAs, and miRNAs, respectively. However, the analysis on lncRNAs is comparatively complex compared with miRNAs or the coding RNAs. As a result, detecting the associations of mRNAs and/or miRNAs can efficiently and accurately illustrate the possible lncRNA functions.

GO functional annotations and KEGG enrichment were carried out for assessing the functions of related DEGs. Besides, according to GO analysis, many related genes were associated with nuclear, nucleoplasm, and nucleolus locations, transcription, and biological regulation. Moreover, most genes were associated with the MF of protein binding, which suggested that they played important part in gene modulation at transcriptional level. At the same time, KEGG enrichment revealed that DEMs focus on some signal pathways, like the PI3K-Akt signaling pathway and Ras pathways.

Proliferation of smooth muscle cells and intimal hyperplasia can be frequently seen during GSV progression, even though atrophic areas are seen [18, 19, 20]. Additionally, GSVs are associated with the transition of smooth muscle cells from contractile phenotype to synthetic one, which indicated that VSMCs are dedifferentiated in GSV pathogenic mechanism [21]. The PI3K/Akt signal transduction pathway exerts an important part in the stability and development of blood vessels, which is tightly related to the development of vascular network [22]. It has been widely suggested that the PI3K/Akt signal transduction pathway relates to VSMC migration and proliferation [23, 24]. For instance, miR-145 mitigated the Hcy-mediated phenotype transition, migration and proliferation of VSMCs via suppressing the PI3K/Akt/mTOR pathway [25]. This study suggested that genes associated with the ceRNA theory function to modulate GSVs via the PI3K/Akt signal transduction pathway.

Thereafter, subnetwork and topological analyses were performed based on the numbers of relation pairs and hub genes. Generally speaking, the lncRNA network with a greater number of relation pairs suggested that lncRNA is the hub exerting vital parts in network structure. According to our present results, lncRNAs AC114730, AC002127, and AC073342 were the key nodes in topology, which had markedly increased lncRNA-miRNA/miRNA-mRNA pair numbers and node degrees relative to additional lncRNAs.

This study also determined all node degrees within the ceRNA network by the cytoHubba plug-in Cytoscape. As a result, the 10 most significant nodes were shown as follows: miR-17-5p, miR-129-5p, miR-1297, miR-20b-5p, miR-33a-3p, miR-27a-3p, miR-301b-3p, miR-24-3p, miR-137, and miR-23b-3p. It is of great significance to explore disease-related miRNAs as well as the corresponding targets for understanding their functions [26]. Moreover, miRNAs, such as miR-21, miR-146a, and miR-214, are related to VSMC functions. miR-24-3p-3p showed direct repression on eNOS, PAK4, and GATA2 within endothelial cells, thereby suppressing blood vessel formation in the process of development as well as in the process of cardiac infarction. miR-24-3p exhibits wide expression within cardiovascular cells, which suggests its effect on regulating blood vessel formation through targeting vascular mural cells. miRNA-24-3p suppression has been previously suggested to prevent VSMC growth through acting on the Bcl-2-like protein 11 [25].

As a result, findings in the present work helps to establish a potent calculation model for predicting the possible lncRNA-miRNA-disease relationships and selecting the potential lncRNAs/mRNAs associated with GSVs and additional disorders. Findings in the present work shed more lights on the mechanism of miRNAs and lncRNAs within GSVs. We established the mechanism of ceRNA in varicose vein disease model for the first time. At present, there is no miRNA-related data in GEO database. We have successfully predicted some miRNAs through the ceRNA mechanism. Besides, the regulating mechanism of lncRNA-miRNA-target mRNA network should be better investigated. Nonetheless, certain limitations should be noted in the present work. Firstly, because few researches have explored the GSV-related molecular mechanism, just 6 pairs of samples were enrolled (including 6 GSVs and 6 matched uninjured samples), which potentially led to false-positive results. Secondly, when diverse gene IDs were converted from a variety of databases, loss of numerous genes may occur, thus decreasing result accuracy.

To conclude, this study showed the lncRNA and mRNA expression profiles of GSV blood vessel and its control based on microarray analysis. Three novel lncRNAs were effectively detected as diagnostic biomarkers. Furthermore, ceRNA network analyses offer potential therapeutic targets for GSVs.

## Figures and Tables

**Figure 1:** Acquisition of differential genes. (a) Volcano plot showing RNAs with differential expression. Genes with upregulation and downregulation are denoted as light red and light green, respectively. (b) lncRNAs with differential expression within GSVs. (c) mRNAs with differential expression within GSVs. Red and blue boxes stand for genes with upregulation and downregulation, separately. Six replicates were set for every group. ∣log2(fold change, FC) | >1 and adjusted *P* < 0.05 were the thresholds for selection.

**Figure 2:** The ceRNA network for lncRNAs-miRNAs-mRNAs for GSVs. Rectangles, ellipses, and diamonds stand for lncRNAs, mRNAs, and miRNAs denoted as green, blue, and red colors, separately.

**Figure 3:** GO analysis as well as KEGG analysis. (a) GO: biological process terms. (b) GO: cellular component terms. (c) GO: molecular function terms. (d) The enriched KEGG pathways.

**Figure 4:** PPI network and hub genes. (a) The PPI network showing DEGs. Node size indicates degree level, with greater nodes indicating the greater degree. (b) Selection of critical mRNAs in PPI network based on DEM connection degree using R.

**Figure 5:** Critical subnetwork of lncRNAs-miRNAs-mRNAs. (a) The network of lncRNA AC114730-miRNAs-mRNAs. (b) The network of lncRNA AC002127-miRNAs-mRNAs. (c) The network of lncRNA AC073342-miRNAs-mRNAs. lncRNAs, miRNAs, and mRNAs are denoted in green, red, and blue colors, separately.

**Figure 6:** Critical subnetworks of lncRNAs-miRNAs-mRNAs. (a) lncRNA-miR-17-5p-mRNA subnetwork. (b) lncRNA-miR-1297-mRNA subnetwork. (c) lncRNA-miR-129-5p-mRNA subnetwork. (d) lncRNA-miR-33a-3p-mRNA subnetwork. (e) lncRNA-miR-20b-5p-mRNA subnetwork. Dark green, light green, and blue nodes represent lncRNAs, miRNAs, and mRNAs, respectively.

**Table 1:** The ranking of lncRNA.

node_name	MCC	EPC	BottleNeck	Closeness	Radiality	Betweenness
AC114730	19	40.843	17	93.08333	4.5404	7323.508
AC073342	11	31.275	18	80	4.14646	3116.466
AC002127	10	35.171	15	81.33333	4.21717	2120.41
AC106875	6	22.218	7	65.03333	3.62121	555.1917
AC002383	6	19.922	3	63.41667	3.56061	456.2976
HHATL-AS1	3	14.266	1	61.26667	3.4899	70.38024
AC079790	3	12.202	4	60.31667	3.4697	201.5566
AP001439	3	7.753	1	54.65	3.11616	70.5266
BACH1-IT3	2	8.611	3	57.08333	3.28788	47.45505
MID1IP1-AS1	1	8.407	1	57.93333	3.35859	0
OOEP-AS1	1	6.033	1	52.23333	2.95455	0
AP002490	1	7.203	1	57.93333	3.35859	0

**Table 2:** The ranking of miRNA.

node_name	MCC	Degree	Closeness	Betweenness
hsa-miR-17-5p	35	35	91.15	6458.953
hsa-miR-1297	25	25	86.8	4896.51
hsa-miR-129-5p	25	25	86.3	5273.315
hsa-miR-33a-3p	23	23	86.21667	5057.459
hsa-miR-20b-5p	20	20	78.7	1561.414
hsa-miR-301b-3p	16	16	78.5	2135.698
hsa-miR-27a-3p	16	16	82.83333	2708.564
hsa-miR-24-3p	15	15	79.08333	2673.176
hsa-miR-137	15	15	75.11667	2360.844
hsa-miR-23b-3p	14	14	76.65	2420.549

## Data Availability

The data of this study are available via GEO database, (https://www.ncbi.nlm.nih.gov/geo/).
